The article "The Impact of Reviewers' Creditworthiness on Consumers' Purchase Intention in Edge Path: Implications for the Coronavirus Disease 2019 Pandemic" was published in 2020. Journal: Front Public Health.

# The Impact of Reviewers' Creditworthiness on Consumers' Purchase Intention in Edge Path: Implications for the Coronavirus Disease 2019 Pandemic

**DOI:** 10.3389/fpubh.2020.619263

**Published:** 2020-12-10

**Authors:** Chen Limei, Liu Wei

**Affiliations:** ^1^School of Management, Nanjing University of Posts and Telecommunications, Nanjing, China; ^2^Department of Finance, Nanjing University of Science and Technology, Nanjing, China

**Keywords:** COVID-19 pandemic, elaboration likelihood model, reviewers' creditworthiness, conformity behavior, purchase intentions

## Abstract

Reviewers' creditworthiness is an important edge clue in the elaboration likelihood model (ELM). This paper takes the online travel booked by consumers as an example and uses the questionnaire data of 417 outbound passengers from Guangzhou Baiyun International Airport. The paper examines the influence of reviewers' creditworthiness on consumer purchase intentions in the edge path through a mediated moderation model. Investigate the mediating role of conformity behavior can influence the reviewers' creditworthiness on purchase. Thus, it examines the moderating effect of consumer involvement. The results show that the degree of consumer involvement moderates the relationship between reviewers' creditworthiness, and the purchase intention is achieved through the mediation of conformity behavior. The higher the degree of consumer involvement, the less impact the reviewers' creditworthiness has on conformity behavior, and the weaker the positive effects of its purchase intention are found. Implications for the coronavirus disease 2019 (COVID-19) era are also discussed.

## Introduction

With the advent of the coronavirus disease 2019 (COVID-19), enterprises are facing an increasing uncertainty shock and networked environment. The World Health Organization (WHO) declares that the new coronavirus may have infected about one in 10 people worldwide, 35 million cases are reported in more than 213 countries, and about 1,080,000 deaths are declared until October 2020 (1). During the COVID-19 period, people spend more time at home, watching reviews and online purchase, rather than off-line purchase; they spend much significant amount of time writing online reviews and are involved more interactively. Motivated by this issue, in this paper, we investigate how to acquire and maintain sustainable marketing management advantages in the uncertain environment of high network interconnection, which has become the research focus of management.

Online comment is one of the important channels for consumers to obtain product or service information, especially in the COVID-19 period. It generally refers to potential or actual customer comments on a product or service published on the Internet (2). As an important social interaction medium, online commentary has become an important factor in establishing an immersive and highly engaged online customer relationship, which in turn affects purchase intention. Credential credibility, as an important dimension variable for online reviews, can significantly increase consumer willingness. In the past 3 years, Internet-based online commentary has become a hot topic for scholars (3). Consumers tend to think that online reviews published by high-creditworthiness commentators are more useful and reliable, thus affecting consumers' purchase intention. At the same time, the “black box” research on the influence mechanism of online reviewers' creditworthiness on the purchase intention will always be a hot issue in marketing management (4). Besides, consumer involvement as an important feature of customer engagement has become a key variable in marketing research that cannot be ignored. China is in the critical period of pandemic and increasing the degree of Internet. Business models and consumer behavior are constantly innovating. The level of consumer participation and interaction has become a key feature that enterprises must consider when formulating marketing strategies. This study has an important implication for online purchase because everyone stays home during the COVID-19 pandemic.

The article "The Impact of Reviewers' Creditworthiness on Consumers' Purchase Intention in Edge Path: Implications for the Coronavirus Disease 2019 Pandemic" was published in 2020. Journal: Front Public Health.

Because of this, this paper aims to explore the relationship between online reviewer's creditworthiness, conformity behavior, and purchase intention based on the theory of involvement and to use consumer involvement as an adjustment variable of the intermediary link. The main contributions of this paper are as follows: firstly, based on trust theory, the mediating role of conformity psychology in the relationship between credibility and purchase intention of reviewers is examined. This paper applies the theory to the network marketing management research, further enriches the research perspective of the “black box” exploration of marketing management, and provides important inspiration for the development and application of network marketing management in the environment of increasing consumer participation. Secondly, this paper examines the influence of reviewer's creditworthiness on the formation of conformity behavior and enriches the research results of conformity mental antecedent variables. Finally, combined with the specific situation in China, this paper examines reviewers' creditworthiness in different consumer involvement scenarios. The influence of the conformity behavior and the conformity behavior on the purchase intention will change, and it is found that different consumer involvement plays a regulatory role in these two links, thus providing practical feasibility suggestions for the marketing practice of Chinese enterprises.

The article "The Impact of Reviewers' Creditworthiness on Consumers' Purchase Intention in Edge Path: Implications for the Coronavirus Disease 2019 Pandemic" was published in 2020. Journal: Front Public Health.

The rest of the paper is organized as follows. *Literature Review and Hypotheses* reviews the literature and explain the hypotheses of the research. *Research Design and Data* explains the design of the study and data. *Empirical Results* provides the empirical results, and *Conclusion* concludes.

## Literature Review and Hypotheses

### Impact of Commentator Credit on Purchase Intention

Reviewers' creditworthiness refers to the reputation of the reviewer or the degree of consumer trust in the reviewer and the acceptance of the content of the review, including the professional competence and reliability of the reviewer. The professional competence of the reviewer mainly means that the reviewer has a certain field of expertise and background to provide the correct information. The credibility of the reviewer refers to the reputation of the reviewer and the credibility of the comment or a certain status in the network (such as senior members and multiple purchases). Reviewers' creditworthiness has a great impact on the impact of online reviews. Consumers tend to think that online reviews published by high-creditworthiness reviewers are more useful and reliable, thus providing more help to consumers' purchasing decisions.

Most domestic and foreign scholars study reviewers' creditworthiness from the professional competence and reliability of reviewers and study their impact on product sales, consumer purchase intentions, and so on. Senecal and Nantel (5) show that most consumers follow a more reliable source of comments or recommendations, which have a higher reference value. Chen and Dhanasobhon (6) point out that comments made by reputable commentators have a greater impact on sales than other reviews. Forman et al. (7) indicate that the increase in sales of products was related to the prevalence of reviewers' disclosure of identity information. Cheung et al. (8) and Guoqing et al. (9) reveal that reviewers' creditworthiness will affect consumers' trust, which in turn affects consumer purchase intentions. The results of Racherla and Friske (10) also confirm that the professionalism of commentators and the reputation of reviewers are positively affecting the perceived usefulness of comments. Therefore, this paper proposes the following assumptions:

*H*_1_*: Reviewers' creditworthiness is significantly positively correlated with purchase intention*.

### Mediation Effect of Conformity Behavior

Conformity behavior means that the consumer changes his or her evaluation of the product or behavior based on the evaluation of the purchase of others. Due to the virtual nature of the network, consumers do not have to give up their original opinions to make purchase decisions that meet the expectations of others when making online purchases. Although there will be no group pressure, the Internet provides a lot of information about other people's purchase behavior (such as online reviews and sales), which can provide a reference for their purchasing decisions. Many domestic and foreign scholars study conformity behavior by researching the characteristics of online reviews and product sales, which have an impact on purchase intention. Huang and Chen (11) show that consumers make their own decisions by referring to other people's purchase behavior and purchase evaluation when shopping online. Xu et al. (12) use brain imaging technology of neuroscience experiments and event-related potential (ERP) to explore the psychological and neural mechanisms of conflicts caused by consumer congregation and anti-conformity decisions, explaining why the phenomenon of congregation in consumer shopping is so popular. Tsao et al. (13) confirmed that conformity behavior has a positive impact on consumer hotel booking behavior. Some scholars have studied the influence of reviewers' creditworthiness on conformity behavior. Critics with higher credibility often play the role of opinion leaders, can influence the decision-making behavior of the majority, and will lead consumers to make conformity behavior. Therefore, this paper proposes the following assumptions:

*H*_2_*: Conformity behavior plays a mediating role in the relationship between reviewers' creditworthiness and purchase intention*.

The article "The Impact of Reviewers' Creditworthiness on Consumers' Purchase Intention in Edge Path: Implications for the Coronavirus Disease 2019 Pandemic" was published in 2020. Journal: Front Public Health.

### The Regulation of Consumer Involvement

The involved theory suggests that individuals' perceptions of objects based on their inner needs, values, and interests form an individual's motivational state of things. Among them, “object” refers to products, brands, advertisements, promotions, or certain shopping situations that consumers may be involved in (14). Sources are used as the criteria for classification and are divided into situational involvement and persistent involvement. In the process of purchasing decision making, consumers will have different levels of involvement due to factors such as personal will, external stimuli, and shopping situation. Therefore, this paper further examines that this kind of consumer involvement plays an important role in the influence of reviewers' creditworthiness and conformity behavior on purchase intention. Among them, consumer involvement refers to different levels of participation, using Zhang and Watts (15) to define the concept, specifically referring to different levels of participation.

The article "The Impact of Reviewers' Creditworthiness on Consumers' Purchase Intention in Edge Path: Implications for the Coronavirus Disease 2019 Pandemic" was published in 2020. Journal: Front Public Health.

Under low involvement, consumer attitudes are more affected by the reliability of online communities; Yaping et al. (16) found that in consumers with low involvement, positive comments are more likely to cause impulsive purchase intentions. Based on the above analysis, the lower the consumer involvement, the more inclined to process information through the edge path, reviewers' creditworthiness may be more concerned, and the high-creditworthiness reviewers often act as opinion leaders, which will make consumers produce conformity behavior and influence purchase intentions. Therefore, this paper proposes the following assumptions:

*H3a: Consumer involvement plays a regulatory role in the relationship between reviewers' creditworthiness and conformity behavior; that is, high consumer involvement weakens the relationship between reviewers' creditworthiness and conformity behavior, while low consumption involvement will strengthen the relationship between the two*.

*H3b: The influence of consumer involvement on the relationship between reviewers' creditworthiness and the purchase intention is achieved through the intermediary of the conformity behavior. The higher the consumer involvement, the less influence the reviewers' creditworthiness has on the conformity behavior and the corresponding. The positive impact of purchase intention is weaker*.

According to the research hypothesis proposed above, the theoretical model for establishing this study is shown in Figure 1.

**Figure 1:** Theoretical model.

## Research Design and Data

### Scale Design

The questionnaire is divided into two parts: basic information and measurement scales. All variables are designed from existing literature to ensure the validity of the measurement. Investigate and measure the reliability and validity of the questionnaire firstly, remove or modify the less reliable items to improve the questionnaire, improve the measurement indicators, form a formal questionnaire, and then conduct a large-scale formal investigation according to the requirements of the sampling design. The specific measurement variables and their measurement index system are shown in Table 1.

**Table 1:** Study variable items and sources.

**Variables**	**Indicator system**	**Measurement basis**
Reviewers' creditworthy-ness RR	I think the reviewers know very well about the outbound travel products or services they want to book	(8)
	I think most online reviewers have a high network reputation	
	I think most online reviewers are trustworthy	
	There are many professional reviewers (such as senior members and multiple purchases)	
Consumer involvement CI	To a large extent, I will evaluate online outbound travel products or services	(15)
	It's important for me to get information about outbound travel products or services from comments	
	I will carefully review online reviews when booking outbound travel products or services	
Conformity behavior CB	Many people who evaluate good outbound travel products or services will also buy	(17)
	Seeing that many people book this outbound travel product or service, I will not think about it	
	I will book outbound travel products or services based on the consensus of many people	
Purchase intentions PI	These comments affect whether I am booking the outbound travel product or service	(18)
	These comments have a big impact on my final scheduled outbound travel products or services	
	These comments have changed my attitude toward booking the outbound travel products or services	
	These comments are a great help for my scheduled outbound travel products or services	

The article "The Impact of Reviewers' Creditworthiness on Consumers' Purchase Intention in Edge Path: Implications for the Coronavirus Disease 2019 Pandemic" was published in 2020. Journal: Front Public Health.

### Sample Selection and Data Collection

Taking the customers who intend to book outbound travel products or services online as a research object, we conducted a sample survey at the exit check-in island of Guangzhou Baiyun International Airport. From March 2018 to April 2018, it took 2 months to issue a total of 514 questionnaires. Among them, 417 were valid questionnaires, and the effective rate of the questionnaire was 81.13%.

### Reliability and Validity Analyses

The reliability and validity of the scale were analyzed using the valid questionnaire data collected, and the reliability and validity information of each measurement scale was calculated, as shown in Table 2.

**Table 2:** Reliability and validity of the scale.

**Variable**	**Cronbach α**	**KMO**	**Bartlett's sphericity test**			**Cumulative total variance**
			**Bangla**	**df**	**Sig**.	
Reviewers' creditworthiness (RR)	0.698	0.735	272.946	6	0.000	52.682%
Consumer involvement (CI)	0.604	0.630	131.546	3	0.000	55.859%
Conformity behavior (CB)	0.588	0.633	117.357	3	0.000	54.841%
Purchase intentions (PI)	0.733	0.744	342.353	6	0.000	55.887%

*KMO, Kaiser–Meyer–Olkin*.

Table 2 shows that the Cronbach α of each scale is >0.58, and the total variance of the cumulative interpretation is above 50%, indicating that the questionnaire has certain credibility in the study. The results of the confirmatory factor analysis using Mplus were chi-square = 183.392, comparative fit index (CFI) = 0.929, Tucker–Lewis index (TLI) = 0.909, and root mean square error of approximation (RMSEA) = 0.062. According to the usual fitting index evaluation criteria, the model fits well, indicating that the research measurements are four independent variables.

The article "The Impact of Reviewers' Creditworthiness on Consumers' Purchase Intention in Edge Path: Implications for the Coronavirus Disease 2019 Pandemic" was published in 2020. Journal: Front Public Health.

### Descriptive Statistical Analysis

The average value, standard deviation, and correlation coefficient between each measured variable are calculated, as shown in Table 3.

**Table 3:** Descriptive statistics and correlation coefficients.

**Variable**	**Mean**	**SD**	**Reviewers' creditworthiness**	**Consumer involvement**	**Conformity behavior**	**Purchase intentions**
Reviewers' creditworthiness	5.294	0.827				
Consumer involvement	5.628	0.841	0.549^***^			
Conformity behavior	5.625	0.815	0.427^***^	0.539^***^		
Purchase intentions	5.454	0.842	0.628^***^	0.635^***^	0.535^***^	

*** *p < 0.001*,

** *p < 0.01*,

* *p < 0.05*.

Table 3 shows that reviewers' creditworthiness, conformity behavior, and purchase intention are significantly and positively correlated, indicating that they are all factors affecting purchase intention. Reviewers' creditworthiness is significantly positively correlated with the conformity behavior and purchase intention, indicating that the conformity behavior maybe is a mediator variable between reviewers' creditworthiness and purchase intention. These results provide the necessary preconditions for analyzing the relationship between reviewers' creditworthiness, conformity behavior, and purchase intentions.

## Empirical Results

### Intermediary Adjustment Effect Model Test

When the direction and size of the relationship between two variables depend on the third variable, there is a regulatory effect. If the modulating effect is to influence the dependent variable through the mediator variable, it becomes an intermediary regulatory effect. According to Fairchild and MacKinnon (19), the regression test procedure for the mediation mode effect model is as follows:

Regression of purchase intentions to reviewer's creditworthiness, consumer involvement, and reviewers' creditworthiness and consumer involvement is shown as follows:

(1) $$\begin{array}{r} \text{Y}={\text{c}}_{0}+{\text{c}}_{1}\text{X}+{\text{c}}_{2}\text{U}+{\text{c}}_{3}\text{XU}+{\text{e}}_{1} \end{array}$$

Among them, Y is purchase intention, X is reviewers' creditworthiness, U is the consumer involvement, XU is the interaction term between reviewers' creditworthiness and the degree of consumer involvement, and e_1_ is the residual regression term. If the coefficient c_3_ of XU is significant, it indicates that the adjustment effect is significant. If the coefficient c_3_ of XU is not significant (the adjustment effect is not significant), it is not necessary to test whether the “mediated effect” is significant.

Regression of the interaction between the conformity behavior, reviewers' creditworthiness, the consumer involvement, and reviewers' creditworthiness and the consumer involvement is shown as follows:

(2) $$\begin{array}{r} \text{W}={\text{a}}_{0}+{\text{a}}_{1}\text{X}+{\text{a}}_{2}\text{U}+{\text{a}}_{3}\text{XU}+{\text{e}}_{2} \end{array}$$

Among them, W is a conformity behavior, X is reviewers' creditworthiness, U is the consumer involvement, XU is the interaction term between the reviewer's creditworthiness and the consumers' involvement, and e_2_ is the regression residual.

The article "The Impact of Reviewers' Creditworthiness on Consumers' Purchase Intention in Edge Path: Implications for the Coronavirus Disease 2019 Pandemic" was published in 2020. Journal: Front Public Health.

Regression of the interaction between reviewers' creditworthiness, the conformity behavior, the consumer's involvement, reviewers' creditworthiness and the consumer's involvement, and the interaction between the conformity behavior and the consumer's involvement is shown as follows.

(3) $$\begin{array}{r} \text{Y}=\text{ c}\prime_{0}+\text{c}\prime_{1}\text{X}+\text{c}\prime_{2}\text{U}+\text{c}\prime_{3}\text{XU}+{\text{b}}_{1}\text{W}+{\text{b}}_{2}\text{WU}+{\text{e}}_{3} \end{array}$$

Among them, Y is purchase intention, X is reviewers' creditworthiness, U is the consumer involvement, XU is the interaction term between the reviewers' creditworthiness and the consumer's involvement, W is the conformity behavior, and WU is the conformity behavior. The consumer enters the interaction term of the two, and e_3_ is the residual regression term. If at least one of the coefficients a_3_ and b_1_, a_3_ and b_2_, and a_1_ and b2 is significant, it indicates that an intermediate adjustment model is established. If c′_3_ is significant, it means that the regulatory effect is partially intervened, and if c′_3_ is not significant, then the regulatory effect affects the dependent variable entirely through the mediator variable.

If the coefficients a_3_ and b_1_, a_3_ and b_2_, and a_1_ and b_2_ are not significant, do bootstrap or Markov chain Monte Carlo (MCMC) interval test. If at least one interval does not contain 0, then an intermediary adjustment model is established; if all three intervals contain 0, then the mediation adjustment model does not hold. This paper uses Mplus7.0 to perform hypothesis testing using the above procedure proposed by Fairchild and MacKinnon (19).

### The Regulatory Role of Consumer Involvement

According to the above test procedure, the adjustment effect of the consumer involvement degree is first tested. Establish a relationship model between reviewers' creditworthiness, consumer involvement, and the interaction between the two and the purchase intention. The results are illustrated in Figure 2.

**Figure 2:** Test of the adjustment effect of consumer involvement.

Since the model is a saturated model, chi-square = 0, df = 0, CFI = 1.000, TLI = 1.000, RMSEA = 0.000, and standardized root mean square residual (SRMR) = 0.000, the model fits well. As can be seen from Figure 2, reviewers' creditworthiness significantly predicts the purchase intention (c_1_ = 0.428, *t* = 10.948, *p* = 0.000), assuming H_1_ is verified. The interaction between reviewers' creditworthiness and the consumer involvement has a significant effect on the purchase intention (c_3_ = −0.134, *t* = −3.611, *p* = 0.000), indicating that the consumer involvement is in reviewers' creditworthiness. Play a regulatory role in the influence of purchase intention, assuming H_3_a is verified.

The article "The Impact of Reviewers' Creditworthiness on Consumers' Purchase Intention in Edge Path: Implications for the Coronavirus Disease 2019 Pandemic" was published in 2020. Journal: Front Public Health.

Figure 3, obtained from the simple slope analysis, reflects the impact of reviewers' creditworthiness and purchase intention for consumers with different degrees of involvement. As can be seen from Figure 3, compared with consumers with high involvement, the value of the reviewers' creditworthiness has a greater regression slope on purchase intention (the regression line is steeper), indicating reviewers' creditworthiness. The same degree of change can trigger a greater degree of change in purchase intention among consumers with low involvement; that is, reviewers' creditworthiness of the low-involvement consumer is more sensitive to changes in purchase intention.

**Figure 3:** The effect of consumer involvement on the relationship between reviewers' creditworthiness and purchase intention.

### Consumer Involvement Has an Intermediary Role in Regulation

Construct a relationship model between the purchase intention, the reviewers' creditworthiness, the conformity behavior, the consumer involvement, the commenter's credibility and the consumer's involvement, and the interaction between the conformity behavior and the consumer's involvement. The test results are shown in Figure 4.

**Figure 4:** Adjustment effect of mediation of consumer involvement.

The fitting indexes of the model are chi-square = 4.307, df = 1, CFI = 0.993, TLI = 0.940, RMSEA = 0.089, and SRMR = 0.012, and the model fits well. The specific model test results are shown in Table 4.

**Table 4:** Results of intermediary effect models.

**Predictor**	(**1**) **(Dependent variable: Purchase intention)**		(**2**) **(Dependent variable: Conformity behavior)**		(**3**) **(Dependent variable: Purchase intention)**	
	**Standard regression coefficient**	***p*-value**	**Standard regression coefficient**	***p*-value**	**Standard regression coefficient**	***p*-value**
Reviewers' creditworthiness	c_1_ = 0.428	0.000	a_1_ = 0.212	0.000	c′_1_ = 0.400	0.000
Consumer Involvement	c_2_ = 0.348	0.000	a_2_ = 0.379	0.000	c′_2_ = 0.272	0.000
Reviewers' creditworthiness × Consumer involvement	c_3_ = −0.134	0.000	a_3_ = −0.111	0.012	c′_3_ = −0.154	0.001
Conformity behavior					b_1_ = 0.196	0.000
Conformity behavior × Consumer Involvement					b_2_ = 0.064	0.158

Table 4 shows that the reviewers' creditworthiness significantly positively predicts conformity behavior (a_1_ = 0.212, *t* = 4.371, *p* = 0.000). The predictive effect of conformity behavior on purchase intention is also significant (b_1_ = 0.196, *t* = 4.946, *p* = 0.000), and reviewers' creditworthiness has a significant direct effect on the purchase intention (c′_1_ = 0.400, *t* = 9.948, *p* = 0.000), indicating that the conformity behavior plays a part in the process of reviewers' creditworthiness affecting his purchase intentions. With role, H2 is verified. At the same time, the interaction between reviewers' creditworthiness and the consumer involvement has a significant predictive effect on the conformity behavior (a_3_ = −0.111, t = −2.509, p = 0.012 < 0.05), and the conformity behavior has a significant predictive effect on the purchase intention (B_1_ = 0.196, t = 4.946, p = 0.000); the interaction term between the conformity behavior and the consumer involvement degree has no significant effect on the purchase intention (b_2_ = 0.064, t = 1.411, p = 0.158 > 0.05). It shows that the adjustment effect of consumer involvement on the relationship between reviewers' creditworthiness and purchase intention is realized through the intermediary of conformity behavior; that is, consumer involvement plays an intermediary role, and H3b is verified. Because the interaction between reviewers' creditworthiness and the consumer involvement is directly predictive of the purchase intention (c′_3_ = −0.154, t = −3.305, p = 0.001), the adjustment effect has some mediation. The adjustment effect of consumer involvement on the relationship between reviewers' creditworthiness and purchase intention is partly achieved through the intermediary of conformity behavior.

The article "The Impact of Reviewers' Creditworthiness on Consumers' Purchase Intention in Edge Path: Implications for the Coronavirus Disease 2019 Pandemic" was published in 2020. Journal: Front Public Health.

Figure 5, which is obtained by simple slope analysis, more clearly shows how reviewers' creditworthiness and consumer involvement interact to influence conformity behavior. As can be seen from Figure 5, compared with consumers with high involvement, the value of the reviewers' creditworthiness to the conformity behavior is larger (the regression line is steeper), indicating reviewers' creditworthiness. The same degree of change can trigger a greater change in conformity behavior in low-involvement consumers; that is, the credibility of the low-involvement consumer is more sensitive to changes in conformity behavior.

**Figure 5:** The effect of consumer involvement on reviewer's creditworthiness and conformity behavior.

The mediation regulation model shows that the adjustment effect of consumer involvement on the relationship between credibility and purchase intention of the reviewer is realized through the intermediary of the conformity behavior. The higher the consumer involvement, the more the influence of reviewers' creditworthiness on the conformity behavior. So the corresponding positive impact on their purchase intentions is weaker.

## Conclusion

In the process of the influence of the reviewers' creditworthiness of the edge path on the purchase intention of the consumer, the adjustment effect of the consumer involvement degree on the relationship between reviewers' creditworthiness and the purchase intention is partially realized through the intermediary of the conformity behavior, that is, the consumer involvement degree. There is an intermediary adjustment between the reviewers' creditworthiness and the purchase intention relationship. The higher the consumer involvement, the less influence the reviewers' creditworthiness has on the conformity behavior, and the weaker the positive influence on the purchase intention. This issue is because, at the high level of involvement, people are more motivated to make the necessary cognition and effort to comment on the information and will extensively search for information and carefully process and evaluate the information, which is the possibility of fine processing of the information. Sex increases, and thus the more inclined to choose the central path, the information content itself has a greater impact on the recipient's attitude. In the case of low involvement, the consumer's processing motivation and processing ability are low. Consumers will choose the edge path to process the information, which will take less time and effort to evaluate the information. The purchase behavior will often be affected by some edge clues (such as reviewer's creditworthiness), and it is more likely to occur in a conformity behavior, thus affecting their purchase intentions.

The relevant conclusions of this study can provide some meaningful revelations and implications for the enterprises in the COVID-19 period: firstly, with the advent of the pandemic, customers spend more time online and acquire more product information online, and we should pay attention to the evaluation system of reviewers' creditworthiness. In the edge path of consumers processing online comment information, reviewers' creditworthiness is an important edge clue. The enterprises can establish a consumer-level membership mechanism, or record the purchase experience of the consumer, and implement an evaluation mechanism for the published online comment. That is, others can like to praise or evaluate online reviews, thus establishing a good evaluation system for reviewers' creditworthiness. Secondly, the enterprises can distinguish customers into different groups since more and more people go shopping online in the period of the COVID-19 by dividing consumers into high-involvement or low-involvement consumers according to the consumer's past purchase experience, published comments, and other information and can adopt corresponding marketing strategies.

The article "The Impact of Reviewers' Creditworthiness on Consumers' Purchase Intention in Edge Path: Implications for the Coronavirus Disease 2019 Pandemic" was published in 2020. Journal: Front Public Health.

Given that people will spend more time at home, watching reviews and online purchase, rather than off-line purchase, they will spend much significant amount of time writing online reviews and be involved more interactively. Therefore, the implication during pandemics is that the weaker positive effects of its purchase intention will persist. Future papers can focus on how re-openings after the COVID-19 pandemic can affect online shopping.

## Data Availability Statement

The raw data supporting the conclusions of this article will be made available by the authors, without undue reservation.

## Ethics Statement

The studies involving human participants were reviewed and approved by The survey in the study has been approved by the ethics committee of Nanjing University of Posts and Telecommunications. The patients/participants provided their written informed consent to participate in this study.

## Author Contributions

CL: data curation, writing—original draft preparation, and visualization. LW: conceptualization, investigation, software, and writing—original draft preparation. All authors contributed to the article and approved the submitted version.

## Conflict of Interest

The authors declare that the research was conducted in the absence of any commercial or financial relationships that could be construed as a potential conflict of interest.
